# Efficacy Evaluation of Neoadjuvant Chemotherapy in Breast Cancer by MRI

**DOI:** 10.1155/2022/4542288

**Published:** 2022-08-04

**Authors:** Yongguang Liu, Mingxiang Wu, Wenyong Tan, Jingshan Gong, Jie Ma

**Affiliations:** ^1^Radiology Department, Shenzhen People's Hospital, Shenzhen 518020, China; ^2^Shenzhen Hospital of Southern Medical University, Shenzhen 518000, China

## Abstract

Breast cancer is a highly harmful malignancy, which often causes great distress to patients and seriously affects their physical and mental health. Breast cancer causes patients to experience decreased appetite, decreased eating, and indigestion, which in turn leads to malnutrition, body wasting, resistance, immune compromise, progressive anemia, cachexia, and, as a result, severe secondary infections. To investigate the efficacy evaluation of neoadjuvant chemotherapy in breast cancer by MRI, forty-eight subjects treated at the hospital from June 2014 to August 2019 were recruited. After the neoadjuvant chemotherapy, the patients were divided into two groups based on the results of histopathological examination, namely, the ineffective group (*n* = 14) and the effective group (*n* = 34). Changes in MRI indicators were compared between the two groups before and after the neoadjuvant chemotherapy. The maximum diameter of lesions decreased significantly after the neoadjuvant chemotherapy than before. The apparent diffusion coefficient (ADC) increased considerably, and the time-intensity curve (TIC) showed a transition from type III to type II/I and from type II to type I. MRI can indicate the maximum diameter of the breast cancer lesion, ADC, and TIC type. Therefore, it can be used to evaluate the efficacy of neoadjuvant chemotherapy for breast cancer and be widely applied in clinical practice.

## 1. Introduction

Breast cancer is the most common cancer in females worldwide. It is not only a local lesion but also, more importantly, a systemic disease. Globally, North America and northern Europe are high incidence areas for breast cancer, southern Europe and South America are middle incidence areas, and most Asian and African countries are low incidence areas. Morbidity and mortality rates are higher in domestic coastal megacities than in inland areas. In terms of urban-rural distribution, the incidence rate was higher in urban than rural areas. The regional distribution of breast cancer mortality is largely consistent with incidence, with high mortality areas remaining in Europe and North America, where the incidence of breast cancer has increased in recent years, and the incidence of breast cancer has increased in all age groups. Our country is also the northern region has a higher incidence of breast cancer than the southern region. Population distribution breast cancer predominates in women and is rare in men, with only about 1 in 100 male breast cancers. In adult females in the same age group, it was higher in unmarried females than in married females. The age distribution in our country has a steep increase in the incidence of breast cancer with increasing age after 25 years of age, which is not smooth until around menopause and can slightly decrease after menopause. Prevalence trends of breast cancer incidence, by the trend of breast cancer incidence to progress toward younger age, breast cancer will become a common disease.

Neoadjuvant chemotherapy (NAC) refers to systemic chemotherapy delivered before local surgery or chemotherapy. This therapy aims to reduce the tumor size and kill cancer migrating to distant organs [1]. Neoadjuvant chemotherapy has become a standard treatment regimen for locally advanced breast cancer. Unfavorable tumor size influences the treatment of breast conservation, while NAC can increase the chance of breast conservation [2, 3]. Besides, patients' responsiveness to neoadjuvant chemotherapy can help predict chemosensitivity, thereby guiding the subsequent treatment for breast cancer [4, 5]. Thus, efficacy assessment of neoadjuvant chemotherapy facilitates clinical treatment of breast cancer. Magnetic resonance imaging (MRI) is a common examination method for breast cancer and is already used to assess chemotherapeutic efficacy for breast cancer [6]. MRI is used to accurately measure the size of breast tumors and detect the presence of multicentric lesions. Compared with mammography and ultrasound, the value of MRI in the determination of the actual size of breast tumors is widely recognized [7, 8]. At present, many studies have proved that MRI has higher sensitivity than conventional imaging for the detection of multiple lesions and multicenter lesions [9].

For some patients suspected of suffering from breast cancer, a breast magnetic resonance examination can be considered. Breast tumors can be found at the same time as magnetic resonance examination [10]. If the shape is irregular, the edge is unclear, or there are burr-like manifestations, some signs of fast in and fast out can be shown during enhancement scanning, and some patients can show slow enhancement. The patients with breast cancer showing obvious enhancement, with obvious burrs of different lengths at the edges, homogeneous or heterogeneous, and irregular ring enhancement of tumors, highly suggest some manifestations of breast cancer [11, 12]. After finding the above signs, it is necessary to further improve the pathological examination, such as extracting certain pathological tissues through the puncture, and determining whether the patient is breast cancer through pathology. After the diagnosis of the patient's breast, we need to formulate a standardized diagnosis and treatment plan according to the patient's physical state, pathological stage, molecular typing, and so on. In this study, we recruited 48 breast cancer patients and evaluated the efficacy assessment of neoadjuvant chemotherapy by MRI.

Breast cancer is a common malignancy in females, and the incidence rate of breast cancer has increased significantly in recent years [13–15]. Neoadjuvant chemotherapy is a good choice for locally advanced and unresectable liver cancer. Neoadjuvant chemotherapy can convert the locally advanced and unresectable liver cancers into resectable ones, achieving downstaging and reducing the distant metastasis rate. The breast conservation rate increases mildly in most resectable tumors (from 7% to 12%), while the recurrence and mortality of breast cancer are reduced [16, 17]. Previous studies have shown that the patients achieving a pathologic complete response (pCR) after neoadjuvant chemotherapy have significantly prolonged overall survival (OS) and disease-free survival (DFS), which is especially true for triple-negative and HER2-positive breast cancers [18]. However, after neoadjuvant chemotherapy, the lesions narrowed and blurred the original images of the breast and axilla. Therefore, the primary breast cancer and axillary lymph node metastasis need to be evaluated in detail before and after neoadjuvant chemotherapy [19]. MRI is an essential tool used to assess tumor scope and treatment responsiveness. Due to the assessment of breast cancer and its different morphologies, MRI is suitable for the phenotypic classification of breast cancer. MRI has a high resolution for soft tissues, and the breast structure can be well indicated [20]. pCR can also be predicted by radiography. Studies have shown that ADC changes are correlated with pCR. On this basis, we can determine whether the patients achieve pCR based on ADC values detected by MRI [21].

Neoadjuvant chemotherapy (NAC) for breast cancer is a part of neoadjuvant systemic treatment (NST) [22]. NST also includes neoadjuvant endocrine therapy and neoadjuvant therapy combined with biological targeted therapy. NST refers to the systemic treatment of breast cancer before local treatment, so it is also called primary systemic treatment. Synonyms with NAC include preoperative chemotherapy, primary chemotherapy, and induction chemotherapy [23, 24]. Breast cancer is prone to hematogenous dissemination. In the “early” stage of breast cancer, subclinical micrometastasis often occurs around the body, so breast cancer is called “systemic disease” [25]. In recent 30 years, a large number of clinical trials have confirmed that DFS and OS are significantly improved after adjuvant chemotherapy for early breast cancer [26]. From the perspective of clinical practice, surgical resection of LABC is often difficult, especially for inoperable LABC, which is a difficult problem for surgeons for a long time. Breast cancer is sensitive to chemotherapeutic drugs. After chemotherapy, the tumor shrinks and is easy to be removed surgically. Some inoperable breast cancer becomes into the resectable status and brings about the opportunity of surgical treatment [27]. It also creates conditions for breast conserving treatment for patients with large tumors and is unsuitable for breast conserving treatment [28].

We confirmed the good efficacy of neoadjuvant chemotherapy for breast cancer, and MRI indicators before and after neoadjuvant chemotherapy were significantly changed. The tumor size and location were clearly shown by MIR. The lesion diameter and volume decreased significantly in the effective group after neoadjuvant chemotherapy, while ADC increased noticeably. The rise in ADC in the ineffective group might be due to the necrosis of tumor lesions, resulting in a significant reduction in the overall density of cells and hence a massive diffusion of water molecules. Before neoadjuvant chemotherapy, TIC was predominantly of type III. After neoadjuvant chemotherapy, 19 patients had a transition from type III to type II/I TIC, and 10 patients had a transition from type II to type I TIC. The above results demonstrated that MRI was a sensitive tool used to assess efficacy after neoadjuvant chemotherapy, which can accurately show the lesions before and after neoadjuvant chemotherapy.

## 2. General Information and Methods

### 2.1. General Information

Forty-eight breast cancer patients admitted to our hospital from June 2014 to August 2019 were selected. The tumor size was above 1 cm in these patients, and all other indicators were normal. None of them were contraindicated for the contrast-enhanced and plain MRI scans. The patients were aged 24–76 years old, with an average of 45.83 ± 12.05 years. The lesion was 11.0–86.0 mm in the maximum diameter, with an average of 37.88 ± 18.83 mm. All of them received biopsies before chemotherapy. Surgeries were performed after neoadjuvant chemotherapy. The surgically resected tissues were submitted for pathological examination. All patients voluntarily signed the informed consent.

### 2.2. Methods

The chemotherapy regimen includes cyclophosphamide + epirubicin + docetaxel, cyclophosphamide + docetaxel, or epirubicin + docetaxel. The NAC was prescribed for 2 days for each cycle, with an interval of 28 days, a total of 3–6 cycles.

For scanning, a superconductor MRI imaging system imported from Germany was used. The breasts were positioned pendently into the two openings of a dedicated breast coil. MRSI was first performed, followed by a dynamic contrast-enhanced MRI. The contrast agent gadopentetate dimeglumine (0.2 mmol/kg) was injected at a dose of 0.2 mmol/kg, with a normal saline flush.

### 2.3. Observation Indicators

The lesion size and ADC were compared before and after the neoadjuvant chemotherapy. The change of the TIC type was also determined based on clinical criteria.

### 2.4. Statistical Analyses

All statistical analyses were conducted using the SPSS 26.0 software. Count data were expressed as percentages (%) and analyzed by the *χ*^2^ test. Measurement data were expressed as mean ± standard deviation (‾*x* ± *s*) and analyzed by *t*-test. *p* < 0.05 indicated a significant difference.

## 3. Results

### 3.1. Lesion Size and ADC Values before and after the Neoadjuvant Chemotherapy

To determine the location and features of lesions, all patients underwent MRI before and after neoadjuvant chemotherapy. The results showed that after neoadjuvant chemotherapy, the maximum diameter of the lesion in the ineffective group decreased significantly (*p* < 0.05), and the ADC value did not increase significantly (*p* > 0.05), as shown in Table 1. In the effective group, the maximum diameter of the lesion decreased significantly (*p* < 0.05), and the ADC value increased significantly (*p* < 0.05), as shown in Table 2.

### 3.2. TIC Types before and after Neoadjuvant Chemotherapy

The blood flow TIC types of tumor lesions were divided into three types, type I (inflow type), type II (plateau type), and type III (outflow type). It has been shown that malignant tumors are mainly of type III or type II and type III curves. MRI results showed that after neoadjuvant chemotherapy, the percentage of patients with type III TIC decreased significantly (*p* < 0.05), while that of patients with type I TIC increased noticeably (*p* < 0.05). There was a transition from type III to type II/I TIC and from type II to type I TIC, as shown in Table 3. MRI was a useful tool to assess the efficacy after neoadjuvant chemotherapy. All MRI indexes were changed, which clearly showed the efficacy after neoadjuvant chemotherapy, as shown in Figure 1. From Figure 1(a), before NAC, T2WI showed a mass in the upper quadrant of the right breast. And in Figure 1(b), after NAC, T2WI showed that the right breast mass was significantly reduced. In Figure 1(c), before NAC, T1W1 was dynamically enhanced. In the early stage, the cross-sectional mass showed a high signal. After NAC, T1W1 dynamic enhancement in the early stage showed that there were small nodular hyperintense signals in the cross section, as shown in Figure 1(d). From Figure 1(e), before NAC, T1W1 demonstrates dynamic enhancement in the late stage showed that the enhancement signal of the mass decreased in the sagittal plane. After NAC, T1W1 dynamic enhancement in the late stage showed a small residual enhancement at the arrow indication in the sagittal plane in Figure 1(f). As can be seen in Figure 1(g), before NAC, the TIC type is type II of the rising platform. However, after NAC, it is the TIC type I of progressive enhancement, as shown in Figure 1(h).

## 4. Discussion

At present, neoadjuvant therapy (NAT) is an important part of comprehensive treatment for breast cancer, and NAT includes neoadjuvant endocrine therapy and targeted therapy with neoadjuvant chemotherapy (NAC), among which NAC is the most widely used. Compared with postoperative adjuvant therapy, neoadjuvant therapy can shrink the tumor and metastatic lymph node volume, stage the primary tumor, and improve the rate of breast conservation. In addition, we can evaluate the sensitivity of tumor to treatment *in vivo*, change the drugs that are not sensitive to the tumor on time and guide subsequent medication, helping clinicians to choose more effective preoperative and postoperative treatment regimens [29]. In recent years, NAT has been gradually promoted and applied in the comprehensive treatment of breast cancer. Evaluation of the efficacy of neoadjuvant treatment for breast cancer is the basis for judging the sensitivity of the tumor to treatment and for developing a plan for the next surgical procedure. Pathological evaluation is the gold standard to objectively reflect the sensitivity of tumors to drug treatment, and a significant histological response suggests that tumors are highly sensitive to therapeutic drugs, but there is a time lag in pathological evaluation. At present, breast imaging is the main method of clinical preoperative evaluation of NAT efficacy, including mammography, ultrasound, and MR examination, and this article focuses on MR examination of the breast [30].

Although breast MR imaging is clearly superior to mammography and ultrasonography for evaluating the efficacy of NAT in breast cancer, its accuracy is also affected to varying degrees by some factors, such as tumor morphology, size, the pattern of regression, heterogeneity of the procedure itself, molecular typing, and treatment options, among which there is again some correlation, and therefore the imaging physician should also fully consider these conditions during evaluation [31].

For the accuracy of breast MR imaging in determining whether a PCR has been achieved after NAT for breast cancer, it was stated that the definition of PCR was defined as the total absence of invasive cancer cells in the breast but the presence of *in situ* cancer components and the absence of tumor cells in the axillary lymph nodes, whereas the evaluation criteria of breast MR imaging were mainly based on the presence of dynamic enhancement, DWI, and the presence or absence of abnormal findings in the breast on MRI, which did not accurately identify the breast cancer as invasive or *in situ*. Therefore, imaging physician and clinicians should also fully recognize this factor affecting the accuracy of breast MRI for predicting PCR after NAT for breast cancer [32].

## 5. Conclusions

In this study, an efficacy evaluation of neoadjuvant chemotherapy in breast cancer by MRI is conducted. Changes in MRI indicators were compared between the two groups before and after the neoadjuvant chemotherapy. The maximum diameter of lesions decreased significantly after the neoadjuvant chemotherapy than before. The ADC increased considerably, and the TIC showed a transition from type III to type II/I and from type II to type I. MRI can indicate the maximum diameter of the breast cancer lesion, ADC, and TIC type. Therefore, it can be used to evaluate the efficacy of neoadjuvant chemotherapy for breast cancer and be widely applied in clinical practice. MRI can facilitate treatment choice in clinical practice.

## Figures and Tables

**Figure 1:** MRI image of triple-negative breast cancer. (a) Before NAC, T2W; (b) after NAC, T2WI; (c) before NAC, T1W1; (d) after NAC, T1W1; (e) before NAC, T1W1; (f) after NAC, T1W1; (g) before NAC, the TIC type; and (h) after NAC, the TIC type is a type I of progressive enhancement.

**Table 1:** Comparison of MRI indicators in the ineffective group before and after neoadjuvant chemotherapy (‾*x* ± *s*).

Time points	Case	Diameter (mm)	ADC (×10^−3^ mm^2^/s)
Before neoadjuvant chemotherapy	14	41.69 ± 22.45	0.914 ± 0.163
After neoadjuvant chemotherapy	14	37.77 ± 22.52	1.031 ± 0.432
t-value		2.24	1.11
*p*-value		0.043	0.287

**Table 2:** Comparison of MRI indicators in the effective group before and after neoadjuvant chemotherapy (‾*x* ± *s*).

Time points	Case	Diameter (mm)	ADC (×10^−3^ mm^2^/s)
Before neoadjuvant chemotherapy	34	36.32 ± 17.25	0.713 ± 0.147
After neoadjuvant chemotherapy	34	18.46 ± 11.91	1.196 ± 0.347
t-value		11.882	9.041
*p*-value		≤0.001	≤0.001

**Table 3:** Comparison of the percentage of patients with different types of TIC cases (%).

Time points	Case	I	II	III
Before neoadjuvant chemotherapy	48	5 (10.4)	18 (37.5)	25 (52.1)
After neoadjuvant chemotherapy	48	26 (54.2)	14 (29.2)	8 (16.7)
*χ* ^2^ statistic		14.226	0.500	8.758
*p*-value		≤0.001	0.480	0.030

## Data Availability

The experiment data used to support the findings of this study are available from the corresponding author upon request.
